RETRACTED

# The Impact of Catalpol on Proliferation, Apoptosis, Migration, and Oxidative Stress of Lung Cancer Cells Based on Nrf2/ARE Signaling

**DOI:** 10.1155/2022/5621341

**Published:** 2022-07-18

**Authors:** Huanyuan Wang, Jingtao Wu, Haiyin Fan, Yuan Ji, Chunbin Han, Chao Li, Sicong Jiang

**Affiliations:** ^1^Department of Thoracic Surgery, Jiangxi Cancer Hospital of Nanchang University, Nanchang, 330029 Jiangxi, China; ^2^Department of Thoracic Surgery, Medical College of Nanchang University, Nanchang, 330006 Jiangxi, China; ^3^Department of Clinical Nursing, Jiangxi Cancer Hospital of Nanchang University, Nanchang, 330029 Jiangxi, China; ^4^Division of Thoracic and Endocrine Surgery, unige.it, 1211 Geneva 4, Switzerland

## Abstract

The effects of catalpol on lung cancer cell proliferation, apoptosis, migration, and oxidative stress via the Nrf2/ARE signaling pathway are investigated in this work. Catalpol-12 g/mL group, catalpol-24 g/mL group, catalpol-48 g/mL group, catalpol − 48 g/mL + vector group, catalpol − 48 g/mL + Nrf2 group, si-NC group, and si-Nrf2 group were used to split lung cancer cells A549 into control groups. Proliferation was detected using the CCK-8 assay; apoptosis was detected using flow cytometry; migration was detected using the transwell chamber; ROS was distinguished using the DCFHDA method; MDA, SOD, and GSH were detected using the microvolume method; and Cleaved Caspase-3, Cleaved Caspase-9, Nrf2, HO-1, MMP-9, and MMP-2 were detected using the Western blot method. Catalpol 12 g/mL and 24 g/mL-48 g/mL treatment decreased the proliferation activity, migration number, and Nrf2, HO-1, MMP-9, and MMP-2 protein levels of lung cancer cells when compared to the control group. SOD and GSH levels of lung cancer cells were decreased, and MDA and ROS levels were increased. Cleaved caspase-3, cleaved caspase-9 protein expression levels, and apoptosis were boosted (*P* < 0.05). The proliferation activity, migration number, and protein levels of Nrf2, HO-1, MMP-9, and MMP-2 in the catalpol − 48 g/mL + Nrf2 group were raised compared to the catalpol − 48 g/mL + vector group, whereas there was an apparent drop in the Cleaved Caspase-3, Cleaved Caspase-9, and apoptosis rate. Similarly, SOD and GSH contents increased, whereas MDA and ROS decreased (*P* < 0.05). The proliferation activity, migration number, and Nrf2, HO-1, MMP-9, and MMP-2 protein levels of lung cancer cells in the si-Nrf2 group were all decreased when compared to the si-NC and control groups. Cleaved Caspase-3 and Cleaved Caspase-9 protein expression, on the other hand, increased as MDA and ROS levels were raised while SOD and GSH levels dropped (*P* < 0.05). It reveals that catalpol inhibits the Nrf2/ARE signaling pathway, which causes antiproliferation, migration, apoptosis, and oxidative stress in cancer cells of lungs. The rate of apoptosis was also lowered.

RETRACTED

## 1. Introduction

Lung cancer is a frequent and common malignant tumor of the respiratory system that has a significant impact on patients' health and quality of life. Biological activities such as lung cancer cell proliferation, migration, and apoptosis are important in lung cancer growth and metastasis [1], which has certain harmful characteristics such as fast development, quite early start, rapid metastasis, and dissemination. It is worth noting that lung cancer cell proliferation, apoptosis, and migration are all linked to tumor growth [2]. Recent research has revealed that [3] nuclear erythroid factor 2-related factor 2 (Nrf2) is a tumor-associated regulatory factor that influences the expression of antioxidant genes including HO-1, oxidative stress, apoptosis, and other processes. Nrf2 may protect cells from external stimuli and promote cell development, as well as can be a key player in the activation of the endogenous antioxidant response. Previous research [4] found that Nrf2 is highly expressed in lung cancer cells, and that downregulating Nrf2 causes apoptosis and oxidative stress in these cells. According to the research, catalpol is an antioxidant, neuroprotective, hypoglycemic, antiaging, anti-inflammatory, and hepatoprotective agent [5]. In previous studies, catalpol has been shown [1, 6–9] to not only suppress tumor development, cell migration, and invasion but also to increase apoptosis in colorectal cancer and gastric cancer cells through modulating signaling pathways. Study shows that catalpol has inhibited the proliferation of bladder cancer cells, breast cancer cells, and nonsmall cell lung cancer cells [10]. According to our findings, the capacity of lung cancer cells to proliferate has reduced, cell apoptosis has raised, and cell migration has decreased following treatment with catalpol. The expression of several components in the cell, including the Caspase protein family, regulates apoptosis which is a process of active cell death [11, 12].

Further, the degradation of the extracellular matrix was one of the primary prerequisites for tumor metastasis [13, 14]. Our findings show that after being treated with catalpol, MMP-2 and MMP-2 protein expression in lung cancer cells decreased, while Cleaved Caspase-3 and Cleaved Caspase-9 protein expression increased. It exhibits more consistency with cell migration and apoptosis detection results, implying that catalpol can induce lung cancer cell apoptosis and inhibit cell migration. Nrf2 is the key regulator of the endogenous antioxidant response. Increased ROS levels can cause Nrf2 to recognize ARE, which leads to the production of antioxidant genes like HO-1 and cell resistance to oxidative stress [15]. Oxidative stress results in a variety of diseases, such as diabetic nephropathy and cerebral infarction [16]. SOD and GSH were antioxidants and decrease in their level results in increase of ROS content that generates a large amount of MDA [17]. Inhibiting Nrf2/ARE might make lung cancer cells more sensitive to chemotherapeutic treatments that cause apoptosis. According to our findings, downregulation of Nrf2 increased the levels of ROS and MDA and decreased the levels of SOD and GSH in lung cancer cells. It also inhibited cell proliferation and migration and promoted cell apoptosis. Lung cancer impacts by suppressing lung cancer growth, migration, and stimulating cell apoptosis, which is a process of active cell death. Catalpol is an iridoid glucoside derived from the dry roots of Rehmannia glutinosa Libosch. It possesses anticerebral ischemia and neuroprotective properties [18]. Catalpol was discovered to block TGF-1, which caused epithelial-mesenchymal transition, invasion, and migration of lung cancer cells in previous studies [10]. However, it is yet uncertain if catalpol influences lung cancer cell growth via modulating Nrf2/ARE signaling. Oxidative stress and Nrf2/ARE signaling have been linked to tumor detection in studies [19–21, 22]. The goal of this study is to see how catalpol affects lung cancer cell proliferation, apoptosis, migration, and oxidative stress through the Nrf2/ARE signaling pathway. It also serves as a reference for the clinical use of catalpol in the treatment of lung cancer.

RETRACTED

## 2. Materials and Methods

The overall experiment is discussed in this section.

### 2.1. Materials

Tongpai (Shanghai) Biotechnology Co., Ltd. provided the human lung cancer cell A549, while Chengdu Dest Biotechnology Co., Ltd. provided catalpol, which had a 20 mg specification and a purity of 98 percent. Beijing Solarbio Technology Co., Ltd. provided the GSH detection kit and the MDA assay kit; Shanghai Yujin Biotechnology Co., Ltd. provided the SOD detection kit; Suzhou Yuheng Biotechnology Co., Ltd. provided the ROS detection kit; Guangzhou Yuanjing Biotechnology Co., Ltd. provided the siRNA control, Nrf2 siRNA, negative control vector (pcDNA), and Nrf2 overexpression vector (pcDNA-Nrf2). Antibodies were bought in the same way. Rabbit anti-Nrf2 antibody was purchased from Abcam in the United States; rabbit anti-Cleaved Caspase-3 antibody and rabbit anti-HO-1 antibody were purchased from Cell Signaling Technology in the United States; rabbit anti-MMP-9 antibody was purchased from Sigma in the United States; rabbit anti-MMP-2 antibody was purchased from GeneTex in the United States; rabbit anti-Cleaved Caspase-9 antibody was purchased from Affinity Biosciences in the United States.

RETRACTED

### 2.2. Methods

#### 2.2.1. Experimental Grouping

Lung cancer cells were separated into many control groups for comparison. “Catalpol-12 g/mL group, catalpol-24 g/mL group, catalpol-48 g/mL group, catalpol-48 g/mL+Vector group, catalpol-48 g/mL+Nrf2 group, si-NC group, and si-Nrf2 group” are among these various groups. The si-NC and si-Nrf2 groups were cells that were transfected with siRNA control and Nrf2 siRNA, respectively. Similarly, the catalpol-12 g/mL group, catalpol-24 g/mL group, and catalpol-48 g/mL group were treated with 12, 24, and 48 g/mL catalpol, respectively. Catalpol − 48 g/mL + vector group and catalpol − 48 g/mL + Nrf2 group were cells transfected with a negative control vector and a Nrf2 overexpression vector, respectively, and then treated with 48 g/mL catalpol. All cells were shifted 24 hours before to the experiment, and catalpol was introduced at 0 hours. A normal grown cell served as the control group. Each group's cells were treated for 24 hours before the follow-up detection. Lung cancer cells were grown in DMEM supplemented with 10% foetal bovine serum. The cell culture temperature was set at 37°C in a 5% CO2 incubator.

#### 2.2.2. CCK-8 Assay to Detect Proliferation

4000 cells and 100 L cell culture medium were introduced to each well after inoculating lung cancer cells into 96-well plates. Catalpol was added at 0, 3, 6, 12, 24, 48, and 96 g/mL, and cells were grouped according to the procedure in Section 2.2.1. After 24 hours of cell culture, 10 liters of CCK-8 working solution were added to each well which were then incubated for 3 hours. Proliferation changes were detected immediately with an enzyme-labeling device, and the results were stated as OD values. The detection wavelength was adjusted to 490 nm.

#### 2.2.3. Western Blot

The cells were collected after being treated according to the technique in Section 1.2.1, and the total protein was extracted using RIPA solution. The BCA kit was used to determine the protein concentration. To promote protein denaturation, boil the protein with 5 × loading buffer for 5 minutes at 100°C. It is electrophoresed using a 10% separation gel and a 5% concentration gel. Add 50 g of protein to each lane, begin electrophoresis at 70 V, and see the blue horizontal line entering the separating gel. Then switch to 100 V and continue electrophoresis until the blue dye reaches the bottom position. The electrophoresis is complete at this point. The NC membrane was activated by immersing it in methanol and then applying a steady current of 250 mA to it for 2 hours. The NC membrane was put in the primary antibody and reacted overnight at 4°C after being blocked with 5% dry skim milk. The NC membrane was then put in the secondary antibody and allowed to bind for 2 hours at room temperature. Since its cost is low, rapidity, wide range of analytes, and minimal background signal, electrochemiluminescence (ECL) is one of several methods used to identify cancer tumors. Electrical potential activates the luminophore in the presence of an activator substance/agent in the (ECL) color rendering process. By fixing the luminophore on the biomolecules, this approach is utilized to quantify the concentration of biomolecules. To put it another way, biomolecules serve as electrical potential carriers for luminophore [21]. The bands' grey values were examined, and the protein expression changes were estimated using GAPDH as a reference. Primary antibodies for Nrf2, HO-1, MMP-9, MMP-2, Cleaved Caspase-3, and Cleaved Caspase-9 were diluted at 1 : 600, 1 : 800, 1 : 1000, 1 : 800, 1 : 1000, 1 : 600, 1 : 800, 1 : 1000, and 1 : 600. Secondary antibodies were diluted at 1 : 4000.

RETRACTED

#### 2.2.4. Flow Cytometry

The lung cancer cells were collected and washed twice with PBS after being treated according to the technique in Section 1.2.1. Finally, about 1106 cells were suspended in 400 liters of binding buffer, to which 5 liters of PI and Annexin V-FITC solution was added and mixed for 15 minutes at room temperature. Add another 100 liters of binding buffer. Flow cytometry can identify it immediately and right away.

#### 2.2.5. Transwell Chamber

A popular test used here was the “transwell chamber migration.” This study explored endothelial cell migration in response to angiogenic inducers or inhibitors. The detection sensitivity of this test is its primary benefit. When it came to lung cancer detection, lung cancer cells were categorized using the procedure described in Section 1.2.1. Suspending the cells in serum-free cell culture medium, the density was altered and adjusted to 1 × 105 cells/200 L. The upper chamber of the transwell chamber received 200 L, while the bottom chamber received 600 L (standard cell culture medium). The cells that could not penetrate the membrane after 24 hours were swept away using a cotton swab. They were stained with crystal violet after being fixed in 90% ethanol (0.1 percent). After that, microscopic observation and count of cell migration were made.

#### 2.2.6. MDA, SOD, GSH, and ROS Detection

The cells were collected after being treated according to the procedure in Section 1.2.1, and the kits were used to determine the amounts of MDA (micro method), SOD (micro method), GSH (micro method), and ROS (DCFHDA method) in the cells. The fluorescence value is given, and the steps are illustrated in the kit.

RETRACTED

### 2.3. Statistical Analysis

The data was analyzed using SPSS25.0. The mean standard deviation (mean SD) is used to express the data. To examine differences across different groups, a one-way ANOVA was employed, with *P* < 0.05 being statistically significant.

## 3. Results

### 3.1. The Effect of Catalpol on the Proliferation of Lung Cancer Cells

As shown in Figure 1, compared with 0 *μ*g/mL, the proliferation activity (OD value) of lung cancer cells treated with 12, 24, 48, and 96 *μ*g/mL catalpol decreased (*P* < 0.05). The survival rate of lung cancer cells treated with 96 *μ*g/mL catalpol was less than 50%, and 12, 24, and 48 *μ*g/mL catalpol were selected for subsequent experiments.

### 3.2. Catalpol Inhibits Nrf2/ARE Signaling in Lung Cancer Cells

When compared to the control group, the protein expression levels of Nrf2 and HO-1 in lung cancer cells in the catalpol-12 g/mL group, catalpol-24 g/mL group, and catalpol-48 g/mL group exhibited a negative trend (*P* < 0.05) (Figure 2).

### 3.3. Inhibition of Nrf2/ARE Signaling on the Proliferation, Apoptosis, and Migration of Lung Cancer Cells

Figure 3 shows that in the si-Nrf2 group, the proliferation activity, migration number, and protein levels of Nrf2, HO-1, MMP-9, and MMP-2 of lung cancer cells decreased, while the expression levels of Cleaved Caspase-3 and Cleaved Caspase-9 and the apoptosis rate raised (*P* < 0.05).

### 3.4. Inhibition of Nrf2/ARE Signaling on Oxidative Stress in Lung Cancer Cells

In Figure 4, in comparison to control group and si-NC group, the contents of MDA and ROS in lung cancer cells in the si-Nrf2 group raised, while the contents of SOD and GSH dropped (*P* < 0.05).

### 3.5. Activation of Nrf2/ARE Signaling Reverses the Effect of Catalpol on the Proliferation, Apoptosis, and Migration of Lung Cancer Cells

Lung cancer cell proliferation activity, migration number, and protein levels of Nrf2, HO-1, MMP-9, and MMP-2 exhibited a declining trend, whereas both protein expressions of Cleaved Caspase-3 and the apoptosis rate showed an increasing trend (*P* < 0.05). The proliferation activity, migration number, and protein levels of Nrf2, HO-1, MMP-9, and MMP-2 in the catalpol − 48 g/mL + Nrf2 group increased compared to the catalpol − 48 g/mL + vector group, while the protein expression level of Cleaved Caspase-3, Cleaved Caspase-9 decreased, and the apoptosis rate also decreased (*P*0.05) (Figure 5).

### 3.6. Activation of Nrf2/ARE Signaling Reverses the Impact of Catalpol on Oxidative Stress in Lung Cancer Cells

The level of SOD and GSH in lung cancer cells in the catalpol-12 g/mL, catalpol-24 g/mL, and catalpol-48 g/mL groups decreased in comparison to the control group, but the amount of MDA and ROS increased (*P* < 0.05). The contents of SOD and GSH in lung cancer cells of catalpol − 48 g/mL + Nrf2 group were raised when compared to catalpol − 48 g/mL + vector group; however, the contents of MDA and ROS were decreased (*P* < 0.05) (Figure 6).

RETRACTED

Figure 6 shows that in comparison with the control group, ^∗^*P* < 0.05. When compared with catalpol-12 *μ*g/mL group, ^#^*P* < 0.05. However, when it is compared with catalpol-24 *μ*g/mL group, ^&^*P* < 0.05. In further comparison with catalpol − 48 *μ*g/mL + vector group, ^△^*P* < 0.05.

## 4. Conclusion

The impact of catalpol on lung cancer cell proliferation, apoptosis, migration, and oxidative stress via the Nrf2/ARE signaling pathway is examined in this work. Proliferation, apoptosis, and migration were detected using the CCK-8 assay, flow cytometry, and transwell chamber, respectively. It is concluded that catalpol increased the levels of ROS and MDA, decreased the levels of SOD and GSH, and downregulated the protein expression levels of Nrf2 and HO-1 in lung cancer cells. Catalpol could induce apoptosis and oxidative stress and inhibit cell proliferation and migration in lung cancer cells via downregulating the activation level of Nrf2/ARE signaling. It provided support for catalpol's antilung cancer mechanism and its clinical use in lung cancer treatment. The in-depth research will also provide new ideas in the prevention and control of breast cancer via catalpol.

## Figures and Tables

**Figure 1:** Proliferative activity of lung cancer cells treated with different concentrations of catalpol. Compared with 0 *μ*g/mL, ^∗^*P* < 0.05.

**Figure 2:** Detection of the expression of Nrf2/ARE signaling proteins Nrf2 and HO-1 in lung cancer cells by Western blot. Note: in comparison to control group, ^∗^*P* < 0.05; in comparison to catalpol-12 *μ*g/mL group, ^#^*P* < 0.05; in comparison to catalpol-24 *μ*g/mL group, ^&^*P* < 0.05.

**Figure 3:** Proliferation, migration, and apoptosis of lung cancer cells after Nrf2 siRNA transfection. Various parts of Figure 3 are further elaborated as below. (a) Cell proliferation activity in lung cancer (OD value). (b) Detection of lung cancer cell apoptosis by flow cytometry. (c) Detection of lung cancer cell migration by transwell chamber (200×). (d) Detection of Nrf2, HO-1, MMP-9, MMP-2, Cleaved Caspase-3, Cleaved Caspase-9, and protein expression in lung cancer cells by western blot; compared with the control group and si-NC group, ^∗^*P* < 0.05.

RETRACTED

**Figure 4:** Contents of MDA, SOD, GSH, and ROS in lung cancer cells transfected with Nrf2 siRNA (^−^*x* ± *s*, *n* = 9). (a) MDA content. (b) SOD content. (c) GSH content. (d) ROS content (relative fluorescence value); compared with the control group and si-NC group, ^∗^*P* < 0.05.

**Figure 5:** The proliferation activity, apoptosis rate, migration number, and protein expression levels. The proliferation activity, apoptosis rate, migration number, and expression levels of protein of Nrf2, HO-1, MMP-9, MMP-2, Cleaved Caspase-3, and Cleaved Caspase-9 in lung cancer cells are transfected with Nrf2 overexpression vector and treated with catalpol. (a) Changes in lung cancer cell proliferation activity (OD value). (b) Detection of lung cancer cell apoptosis changes by flow cytometry. (c) Detection of lung cancer cell migration by transwell chamber (200×). (d) Detection of Nrf2, HO-1, MMP-9, MMP-2, Cleaved Caspase-3, and Cleaved Caspase-9 protein expression in lung cancer cells by western blot; compared with the control group, ^∗^*P* < 0.05; compared with catalpol-12 *μ*g/mL group, ^#^*P* < 0.05; compared with catalpol-24 *μ*g/mL group, ^&^*P* < 0.05; compared with catalpol − 48 *μ*g/mL + vector group, ^△^*P* < 0.05.

**Figure 6:** Contents of MDA, SOD, GSH, and ROS in lung cancer cells after transfection with Nrf2 overexpression vector and catalpol treatment. Various parts of Figure 6 are elaborated as under for better understanding. (a) MDA content. (b) SOD content. (c) GSH content. (d) ROS content (relative fluorescence value).

## Data Availability

Data to support the findings of this study is available upon reasonable request from the corresponding author.
